# Construction and Analysis of Indicators of the Labor Education System Based on the Gray Correlation Degree Model

This article has been retracted.

**DOI:** 10.1155/2022/2281469

**Published:** 2022-08-12

**Authors:** Ling Huang

**Affiliations:** College of Marxism of Hunan Biological and Electromechanical Polytechnic, Changsha 410000, China

## Abstract

Labor education is a complex concept whose value is not only the sum of labor + education. It plays an extremely important role in the growth education of students. Its fundamental purpose is to cultivate students' good technical literacy, improve their practical skills, and form innovative thinking. The monitoring data show that the path of labor education in schools is good, but there are also problems such as unbalanced development of labor practice, insufficient leading role of schools, insufficient basic role of families, and serious lack of social support. Responsibility index, learning motivation, motor health, and self-awareness are significantly and positively correlated with labor practice index. Based on the gray relationship theory, this paper selected relevant data of Chinese students, calculated the comprehensive gray relationship degree between each factor and students' labor reeducation level, and analyzed the variables; the new connotation of education, the construction of labor education evaluation index system, and the construction of labor education support system were studied.

## 1. Introduction

Labor education means organizing students to learn certain technical knowledge of labor and to participate in certain labor activities so that they can acquire the viewpoint of labor, develop labor habits, understand the basic principles of modern production technology, and master the corresponding basic skills so that they can use them in the future [1], engage in educational activities, and lay the foundation for various occupations [2, 3]. The current labor education in colleges and universities can be analyzed from the perspective of colleges and students [3–5]. The following problems exist: lack of labor education courses in colleges and universities and lack of conducting labor education courses as basic courses in universities; but, few schools actually include labor education in their course syllabus [6]. Even if the school reluctantly opens the door to this course and the teacher does not say so, it is painful for both teachers and students to offer this course [7]. Students are not aware of labor education; most students grow up in the context of examinations and still have a utilitarian purpose of education after the university. Students have been immersed in the frenzy of textual research, neglecting the development of their own interests and creative consciousness and lacking the awareness of actively improving their practical skills [8].

From basic education to higher education, we have emphasized the all-round development of students. However, in terms of concrete implementation, we have been following a talent development route that emphasizes achievement at the expense of ability [9]. Labor education is a bridge between students' learning and employment. Students can acquire relevant practical skills through labor education to prepare for their future employment [10–12]. Schools are an important platform for implementing labor education. First, schools should invite vocational and labor education talents to popularize labor education for all teachers so that college teachers can understand labor education objectively and change old concepts [13]. Secondly, schools should cooperate with enterprises and select outstanding talents from enterprises to provide relevant practical courses for students in schools, which can not only enrich students' campus life but also exercise their practical skills and give them a comprehensive understanding of labor education. Finally, schools should develop corresponding labor education bases according to local characteristics, which can not only establish the school brand but also provide students with sufficient training opportunities [14–16].

Labor education is closely related to each of us, and it permeates all aspects of our lives [17].

In this paper, we monitored two aspects: the development of students' labor education in school and at home and students' labor concepts, labor dynamics, and labor habits, including four dimensions of self-service, homework, in-school labor, and out-of-school labor [18]. It can be seen that the gap between urban and rural areas and disciplines is not very large in terms of support for labor education in schools. Urban teachers are slightly higher than rural teachers in counties and villages, and math and science teachers are slightly higher than Chinese teachers. Parents generally believe that labor education can promote the healthy development of their children. When asked if students' participation in labor is a good exercise, 65.2% of parents strongly agreed and 24.4% agreed. Parents are very satisfied with the current state of education in their schools, and 84% of parents say they are relatively satisfied or very satisfied. Also, comparing urban and rural data, there was no significant difference between urban and rural parents [19].

## 2. Gray Relational Analysis

### 2.1. Calculation of Gray Absolute Relevance Degree

First, determine the reference sequence *X*_0_ and the comparison sequence *X*_*i*_ according to the specific problem of the study:

(1) $$\begin{array}{c} X_{0}=\left(x_{0}\left(1\right),x_{0}\left(2\right),\ldots ,x_{0}\left(n\right)\right),\\ X_{i}=\left(x_{i}\left(1\right),x_{i}\left(2\right),\ldots ,x_{i}\left(n\right)\right),\;\left(i=1,2,\ldots ,m\right). \end{array}$$

Next, find the zeroed image of the starting point of the reference sequence and the comparison sequence:

(2) $$\begin{array}{c} X_{0}^{0}=\left(x_{0}^{0}\left(1\right),x_{0}^{0}\left(2\right),\ldots ,x_{0}^{0}\left(n\right)\right)=\left(x_{0}\left(1\right)-x_{0}\left(1\right),x_{0}\left(2\right)-x_{0}\left(1\right),\ldots ,x_{0}\left(n\right)-x_{0}\left(1\right)\right),\\ X_{i}^{0}=\left(x_{i}^{0}\left(1\right),x_{i}^{0}\left(2\right),\ldots ,x_{i}^{0}\left(n\right)\right)=\left(x_{i}\left(1\right)-x_{i}\left(1\right),x_{i}\left(2\right)-x_{i}\left(1\right),\ldots ,x_{i}\left(n\right)-x_{i}\left(1\right)\right). \end{array}$$

Finally, find the gray absolute correlation degree *ε*_0*i*_ of the reference sequence *X*_0_ and the comparison sequence *X*_*i*_:

(3) $$\begin{array}{c} \varepsilon_{0i}=\frac{1+\left|S_{0}\right|+\left|S_{i}\right|}{1+\left|S_{0}\right|+\left|S_{i}\right|+\left|S_{i}-S_{0}\right|}. \end{array}$$

Here,

(4) $$\begin{array}{c} \left|S_{0}\right|=\int_{1}^{n}X_{0}^{0}\text{d}t\\ =\left|\sum_{k=2}^{n-1}x_{0}^{0}\left(k\right)+\frac{1}{2}x_{0}^{0}\left(n\right)\right|,\\ \left|S_{i}\right|=\int_{1}^{n}X_{i}^{0}\text{d}t\\ =\left|\sum_{k=2}^{n-1}x_{i}^{0}\left(k\right)+\frac{1}{2}x_{i}^{0}\left(n\right)\right|,\\ \left|S_{i}-S_{0}\right|=\left|\sum_{k=2}^{n-1}\left(x_{i}^{0}\left(k\right)-x_{0}^{0}\left(k\right)\right)+\frac{1}{2}\left(x_{i}^{0}\left(n\right)-x_{0}^{0}\left(n\right)\right)\right|. \end{array}$$

### 2.2. Calculation of Gray Relative Correlation Degree

First, find the initial value of *X*_0_and *X*_*i*_ as *X*_0_′and *X*_*i*_′:

(5) $$\begin{array}{c} X_{0}^{\prime }=\frac{X_{0}}{x_{0}\left(1\right)}=\left(\frac{x_{0}\left(1\right)}{x_{0}\left(1\right)},\frac{x_{0}\left(2\right)}{x_{0}\left(1\right)},\ldots ,\frac{x_{0}\left(n\right)}{x_{0}\left(1\right)}\right),\\ X_{i}^{\prime }=\frac{X_{i}}{x_{i}\left(1\right)}=\left(\frac{x_{i}\left(1\right)}{x_{i}\left(1\right)},\frac{x_{i}\left(2\right)}{x_{i}\left(1\right)},\ldots ,\frac{x_{i}\left(n\right)}{x_{i}\left(1\right)}\right). \end{array}$$

Next, find the zeroing image of the starting point of *X*_0_′ and *X*_*i*_′.

Finally, find the relative correlation degree *r*_0*i*_ between *X*_0_ and *X*_*i*_.

(6) $$\begin{array}{c} r_{0i}=\frac{1+\left|S_{0}^{\prime }\right|+\left|S_{i}^{\prime }\right|}{1+\left|S_{0}^{\prime }\right|+\left|S_{i}^{\prime }\right|+\left|S_{i}^{\prime }-S_{0}^{\prime }\right|}. \end{array}$$

### 2.3. Finding the Gray Comprehensive Correlation Degree

*ρ*_0*i*_=*θε*_0*i*_+(1 − *θ*)*r*_0*i*_, where *θ* ∈ [0, 1]. (6) is generally acceptable when *θ* = 0.5. If we pay more attention to the relationship between absolute quantities, it can be larger. If you pay more attention to the rate of change, *θ* can be smaller.

## 3. Data Collection

Student labor practice mainly includes on- and off-campus labor organized by the school, as well as student self-service and housework. As shown in Figure 1, the survey found that junior high school students have relatively good on-campus labor practices and weaker off-campus practices, self-service is relatively good, and housework is relatively weak. In terms of self-service and housework, students in private migrant schools are significantly stronger than students in other schools, but there is no significant difference in labor practices inside and outside the school. In different regions and gender dimensions, the labor practices of students are basically similar.

Table 1 further analyzes the students' participation in labor practice activities organized by the school and presents the types and frequencies of students' participation in labor practice both inside and outside the school.

The data show that the frequency of students' on-campus labor practice is relatively high, and the proportion of students participating in on-campus labor practice once a week is 61.8%. Although the types of students' off-campus labor practice are relatively rich, the frequency is generally low. 24.9% of the students have never participated in off-campus labor practice, and less than 20% of the students have participated three or more times. Junior high school should be the initial stage of career experience, and 18.6% of students have participated in career experience activities. In addition, 38.8% and 52.8% of students have participated in “other” on-campus and off-campus labor practices other than the options, respectively, which shows that the types of labor practices are quite diverse.

Junior high school students have strong self-service ability, and 62.1% of the students take the initiative to organize their daily life and school supplies at least three times a week. Junior high school students participate better in housework.  Table 2 presents the frequency of students doing housework in different regions and genders. 40% of students said they do housework at least three times a week, and 39.4% said they do housework once or twice a week. Among the students who do housework every day, towns and villages account for the highest proportion (19.2%). In terms of gender, boys who do housework at least three times a week account for 41.9%, 3.9% points higher than girls. Most of the students who do not do housework are urban students or boys. It can be seen that the participation in housework of rural students in townships and villages is better than that of students in the county and urban areas.

The data in Table 3 show that 5.6% of the students do the “cooking” housework every day on weekends, 26.8% of the students do the “cooking” housework once or twice a month, and 39.4% of the students basically do not do the “cooking” housework.

The monitoring data show that the labor education path of junior high schools in Zhejiang province is sound.  Figure 2 presents school labor education implementation from teacher questionnaires.

As can be seen from Figure 2, among the compulsory courses for labor, technology, and comprehensive practice activities in schools, 1-2 times a week accounted for 30.9% and 1-2 times every two weeks accounted for 17.6%. Schools carry out sanitation, green planting, class activities with the theme of labor education, clubs, interest groups, and other on-campus labor more frequently. In terms of the frequency of teachers organizing students to carry out on-campus labor, 1-2 times a week accounted for 30.2%, at least once a month accounted for 40.2%. The school also offers labor practice expansion elective courses such as housekeeping, cooking, handicraft, and gardening to enrich the course content. The frequency of offering these courses is 1-2 times a week, accounting for 21.9%, and 1-2 times every two weeks, accounting for 14.5%. The school promotes and evaluates the effectiveness of home labor education in the form of homework assignments. The frequency of homework assignments for students is 16.5% once or twice a week and 15.1% is once or twice every two weeks. The frequency of off-campus labor practices such as public welfare activities, voluntary services, research trips with labor education as the theme, and social practice organized by schools is relatively low, accounting for 57.4% once or twice per semester and 9.1% once or twice a week. This shows that although the school can carry out labor practice education normally, its frequency is relatively low and the content is single. It is urgent to build a scientific labor education curriculum system and explore diversified labor education practice paths.

The data in Table 4 show that among teachers who arrange homework once or twice a week, the proportions of urban, county, and township and rural teachers are 18.9%, 16.9%, and 14.5%, respectively. It can be seen that urban teachers' homework assignments are better than county teachers, and county teachers are better than township and rural teachers.

## 4. Results and Analysis

According to the calculation result of the gray correlation degree, the correlation degree of each factor is compared in pairs and the judgment matrix is constructed. Scales 1, 3, 5, 7, and 9 are used to indicate that factor *X*_*i*_ is equally important, slightly important, clearly important, strongly important, and extremely important compared to factor *X*_*j*_, while scales 2, 4, 6, and 8 indicate the difference between the above judgments. After the judgment matrix is constructed, use the following formula to calculate its influence:

(7) $$\begin{array}{c} \lambda_{\text{max}}=\frac{1}{n}\frac{{\left(BW\right)}_{i}}{W_{i}}. \end{array}$$

Here, *λ*_max_ represents the largest eigenvalue of the judgment matrix *B*; *W* represents the normalized eigenvector corresponding to *λ*_max_; *W*_*i*_ represents the influence of the ranking of the constituent factors; and *n* represents the dimension of the judgment matrix *B*. In order to check the consistency of the judgment matrix *B*, the consistency index CI needs to be calculated and the corresponding calculation formula is as follows:

(8) $$\begin{array}{c} \text{CI}=\frac{\lambda_{\text{max}}-n}{n-1}. \end{array}$$

We compare CI with the average random consistency index RI to test whether the judgment matrix B is consistent. For matrices of orders 1 to 16, the values of RI are listed in Table 5.

The first-order and second-order judgment matrices are completely consistent. Starting from order 3, the random consistency ratio of the judgment matrix needs to be calculated: CR=(CI/RI). When CR < 0.1, it is considered that the judgment matrix has satisfactory consistency; otherwise, the judgment matrix is readjusted.

As shown in Table 6, the correlation analysis was made between the labor practice index and monitoring indexes, such as sense of responsibility, learning motivation, sports health, self-cognition, family education, teacher-student relationship, parent-child relationship, hobbies, parent participation, and peer relationship. It shows that there is a significant positive correlation between each monitoring index and the labor practice index and the labor practice index has the highest correlation with the sense of responsibility index.

Responsibility refers to the process by which students take responsibility for themselves, others, collectives, and society by performing certain normative behaviors, including fulfilling obligations, duties, and other requirements. On the one hand, students with a strong sense of responsibility often participate in more labor practices; on the other hand, labor practice activities are just a good carrier to enhance students' sense of responsibility and develop courage and perseverance [20–22].

It can be seen from Figure 3 that with the improvement of the level of responsibility index, the score of labor practice index is getting higher and higher and the two subdimensions also have similar conclusions. The labor practice index scores for each level of “citizen responsibility” are higher than those of “self-responsibility.” It can be seen that the awareness of civic responsibility has a relatively large impact on labor practice.

It can be seen from Figure 4 that with the improvement of family education level, the score of labor practice index is getting higher and higher and the three subdimensions also have similar conclusions. The labor practice index scores corresponding to each level of “democracy and respect” are higher than those of “affirmation and encouragement” and “independence training.” It can be seen that the family education method of “democracy and respect” has a relatively large impact on labor practice.

As can be seen from Figure 5, from the perspective of the relationship between participation in various types of regular on-campus labor practice activities organized by the school and students' sense of responsibility, the scores of students' sense of responsibility index who participated in on-campus activities were much higher than those who did not participate in on-campus activities and participating in vocational postexperience activities was more helpful in the formation of a sense of responsibility.

As can be seen from Figure 6, from the perspective of the relationship between participation in various types of regular off-campus labor practice activities organized by the school and students' sense of responsibility, students who participated in off-campus activities scored much higher than those who did not participate in off-campus activities and participated in community-friendly public welfare services or cultural activities. Publicity activities are more conducive to the formation of a sense of responsibility.

Labor education has the comprehensive educating value of cultivating morality, enhancing intelligence, strengthening body, and nurturing beauty, and it is of great significance to fully tap its hidden value of promoting the healthy growth of students. In fact, labor education must not only be presented at the material level but also must be sublimated at the spiritual level and attention should be paid to cultivating students' labor literacy. For example, in the process of doing housework, students learn to manage their own time, coordinate the relationship between housework and study, and do things in a short time and efficiently. Students undertake housework as much as they can, cultivate their sense of independence and the ability to overcome difficulties, appreciate the hardships of labor, cherish the fruits of labor more, feel the joy of labor, and form a positive attitude towards labor.

## 5. Countermeasures and Suggestions

Based on the monitoring results and the analysis of the current situation of labor education in Zhejiang province, the following three suggestions are put forward for the comprehensive promotion of labor education for junior high school students.

### 5.1. Endowing Labor Education with New Connotation

Monitoring data show that labor education has a positive effect on the formation of students' “responsibility”; some studies have also shown that “responsibility” and “learning motivation” have a significant positive effect on students' academic performance. It can be seen that it is necessary to give the original labor education a new connotation.

It can be seen that in terms of standpoint, it is necessary to fully realize the combination of the “substance” rather than “form” of education and productive labor. In terms of content, it embodies a developmental view of education, emphasizing leisure education and consumer education. In terms of function, it emphasizes labor. The existential value of the individual is to endow the individual with a sense of value and meaning of self-existence in labor education, enrich their relationship attributes, and enhance their aesthetic personality; in practice, it should cultivate students' correct labor concepts and attitudes and build an integrated and open labor education practice system. This kind of labor education focuses on the cultivation of labor literacy and cannot be simply understood as the establishment of labor classes. Morality, intelligence, physique, beauty, and labor mentioned in the educational policy are all concepts of literacy, and they do not correspond to specific disciplines; that is, it cannot be said that “morality” corresponds to the discipline of moral education and “physical” cannot be regarded as a physical education class. In the same way, students' labor literacy is not only cultivated in labor classes but also in the daily care of home and school, the sanitation rotation of the class, the layout of the environment, the physical measurement and field investigation of subject teaching, the practical activities of various comprehensive practice courses and the cultivation function of labor literacy [23, 24].

Junior high school students are in adolescence, and their growing physical maturity prompts them to seek independence psychologically, gradually reduce their dependence on their parents, and hope to get rid of their parents' “control.”

However, they also face many challenges and problems in their studies and life and still need the support, companionship and guidance of their parents. Therefore, parents need to change their educational roles, adjust their parenting methods, give their children trust and understanding, provide timely help and guidance, infiltrate the cultivation of sense of responsibility in labor education, and stimulate children's learning motivation.

### 5.2. Constructing the Labor Education Evaluation Index System

Schools should incorporate labor education into their teaching plans, set up labor courses, cultivate labor literacy, continuously improve labor education programs and security systems, and implement refined labor education evaluations. According to the “opinions,” a labor education evaluation index system with regional characteristics is formulated. For example, curriculum settings generally include labor compulsory courses, labor development courses, labor weeks, and subject penetration. Teaching implementation includes teaching content, teaching form, teaching resources, and teaching evaluation. The guarantee mechanism includes system guarantee, teacher guarantee, funding investment, and safety. Labor literacy includes labor concepts, labor knowledge and skills, labor habits, and labor practice capabilities. Curriculum settings can also draw lessons from mature foreign experience. For example, Japan's labor courses include home economics, lunch education, and field education; Germany's labor courses include technology, economics, home economics, and vocational skills; Finland's labor courses include handicraft, home economics, programming courses, and comprehensive courses.

At the same time, the results of students' usual labor are included in the personal comprehensive quality evaluation and the education supervision department incorporates the results of school labor education into the school's developmental assessment to promote the effective achievement of labor education goals.

### 5.3. Construction of the Labor Education Support System

Labor education must permeate the moral, intellectual, physical, and aesthetic education in schools and cannot be done without the operation and social support of the home and school. Therefore, it is necessary to strengthen the cooperation between school, family, and society to carry out labor education and ensure the effective implementation of labor education. Teachers should make full use of the special activity classroom as the main post to educate students about labor so that they can form correct labor values; they should praise students in the class who love labor and have strong labor skills and encourage other students to follow them. Schools should carry out relevant activities to stimulate students' interest in labor, such as organizing tree planting festivals and small production competitions, which not only help transform passive labor into conscious labor but also improve students' ability to use their hands and brains.

## Figures and Tables

**Figure 1:** Structural characteristics of labor practice of junior middle school students in Zhejiang province.

**Figure 2:** Distribution of school labor practice activities.

**Figure 3:** Responsibility index.

**Figure 4:** Labor practice index scores under different family education levels.

**Figure 5:** Relationship between different types of on-campus labor practices and sense of responsibility.

**Figure 6:** The relationship between different types of off-campus labor practices and sense of responsibility.

**Table 1:** The situation of students participating in labor practice.

School labor practice	Frequency	No	Annually	Once a semester	Once a month	Once a week
		2.4%	1.2%	8.1%	26.7%	61.9%
	Type (multiple choices)	Practice-based learning	Various service posts of the school	Professional postexperience activities	other	
		42.4%	51.6%	18.9%	39.1%	

Off-campus labor practice	Frequency	Never	1∼2 times	3∼6 times	6∼10 times	More than 10 times
		25%	55.4%	16.4%	2.1%	1.5%
	Type (multiple choices)	Community convenience and public welfare services	Cultural publicity activities	Environmental voluntary activities	Caring and serving others	Other
		22.6%	23.4%	32.9%	31%	52.9%

**Table 2:** Frequency of housework for students in different regions and genders in the province.

Whole province		Do it every day (%)	Four times on Wednesday (%)	Twice a week (%)	Once or twice a month (%)	Basically not (%)
		15.6	24.4	39.5	12.4	8.4
Regional nature	City	12.96	22.3	40.4	15.1	9.8
	County town	12.5	22.6	41.5	14.3	8.9
	Rural township	19.3	26.4	37.6	9.8	7.4

Gender	Male	17.3	24.7	36.7	12.2	9.5
	Female	14.1	23.9	42.3	12.6	7.4

**Table 3:** Frequency of students doing “cooking” housework on weekends.

	Never or hardly (%)	Once or twice a month (%)	Once or twice a week (%)	3 or 4 times a week (%)	Every day or almost every day (%)
Whole province	39.5	26.9	22.6	5.7	5.7

**Table 4:** Frequency of homework assignments.

	Never or hardly (%)	Once or twice a month (%)	Once or twice a week (%)	3 or 4 times a week (%)	Every day or almost every day (%)
City	13.12	32.2	21.3	14.8	18.7
County town	16.2	30.2	21.6	15.6	17.1
Rural township	17.9	31.2	21.2	15.3	14.7

**Table 5:** Average stochastic consistency indicators RI.

Orders	1	2	3	4	5	7	8	9	10	11	12	13	14	15	16
RI	0	0	0.53	0.88	1.13	1.25	1.37	1.42	1.46	1.51	1.54	1.57	1.59	1.60	1.62

**Table 6:** Relationship between monitoring index and labor practice index.

Index	Correlation coefficient
Responsibility index	0.352
Learning motivation index	0.278
Exercise health index	0.257
Self-cognition index	0.255
Family education index	0.219
Self-cognition index	0.256
Family education index	0.219
Teacher-student relationship index	0.215
Parent participation index	0.207
Peer relationship index	0.173

## Data Availability

The experimental data used to support the findings of this study are available from the author upon request.
